The article "Clinical Efficacy of Dienogest versus Levonorgestrel-Releasing Intrauterine System for Adenomyosis" was retracted in 2023. Reasons: unreliable results or conclusions; concerns about the data; concerns about the peer review; concerns about the citations.

# Clinical Efficacy of Dienogest versus Levonorgestrel-Releasing Intrauterine System for Adenomyosis

**DOI:** 10.1155/2022/1995472

**Published:** 2022-07-15

**Authors:** Siyuan Yang, Yuchen Liu, Jing Wen, Yi Sun, Fang Ren

**Affiliations:** Department of Gynecology, The First Affiliated Hospital of Zhengzhou University, Zhengzhou, China

## Abstract

**Objective:**

The aim of this study is to evaluate the efficacy of dienogest versus levonorgestrel-releasing intrauterine system (LNG-IUS) for the treatment of adenomyosis.

**Methods:**

In this retrospective study, 85 patients with adenomyosis treated in The First Affiliated Hospital of Zhengzhou University from May 2019 to May 2021 were recruited and assigned, via the random number table method at a ratio of 1 : 1, to receive either dienogest (observation group, *n* = 41) or LNG-IUS (control group, *n* = 44). The patients presented with dysmenorrhea, menorrhagia, and infertility. The treatment outcome was evaluated using visual analogue scale (VAS) scores, menstrual volume, uterine volume, endometrial thickness, and adverse reactions.

**Results:**

After treatment, the VAS score, menstrual volume, and endometrial thickness were significantly decreased in both groups (*P* < 0.05). After 3, 6, and 12 months of treatment, patients receiving dienogest showed significantly lower VAS scores compared to those treated with LNG-IUS (*P* < 0.05). After 6 and 12 months of treatment, patients receiving dienogest were also found to have a significantly better control of menstrual volume compared to those receiving LNG-IUS (*P* < 0.05). Irregular vaginal bleeding was mainly seen in the first 3 months of treatment with dienogest. The incidence of irregular vaginal bleeding lasting more than 6 months was lower with LNG-IUS treatment than with dienogest (*P* < 0.05), and it decreased in both groups as the duration of treatment increased.

**Conclusion:**

Dienogest effectively alleviates dysmenorrhea, relieves pelvic pain, dyspareunia, and reduces menstrual flow in patients with adenomyosis, with few adverse effects and a high safety profile.

## 1. Introduction

Adenomyosis is caused by invasion of the uterine smooth muscle by endometrial glands and stroma, with compensatory hyperplasia and hypertrophy of the surrounding smooth muscle cells. The lesions can be local or diffuse [1]. It typically occurs in women between 30 and 50 years of age. Epidemiological surveys have found that the incidence of the disease is increasing annually [2]. Although the specific mechanism remains unclear, it is speculated to be associated with a large number of births, spontaneous and induced abortions, and endometrial hyperplasia, endometriosis, surgical trauma, cesarean section or curettage, and smoking. Three subtypes of adenomyosis according to MRI findings include the following: (a) diffuse type; (b) focal type; and (c) extrinsic type. The main clinical manifestations of adenomyosis include progressive dysmenorrhea, menorrhagia, chronic pelvic pain, dyspareunia, and infertility. These features severely impact the physical and mental state of patients, and reduce the overall quality of life [3]. Hysterectomy is the mainstay of treatment for adenomyosis [4], and conservative treatment is reserved for patients who refuse to undergo hysterectomy, usually because of fertility reasons [5].

Currently, oral contraceptive/low‐dose estrogen–progestin (OC/LEP), progestins, and gonadotropin‐releasing hormone (GnRH) agonist are controversial. The conservative treatment options include oral dienogest and levonorgestrel intrauterine System (LNG-IUS), both of which are effective at alleviating symptoms and improving the patient's quality of life. LNG-IUS is an intrauterine device that releases progestin locally. It is effective due to progestogenic influences on adenomyosis foci, atrophy of the utopic endometrium and the control of endometrial factors that changed during adenomyosis. Despite its effectiveness [6], it is associated with such side effects as irregular vaginal bleeding, amenorrhea, back pain, excessive vaginal discharge, and dislodgement. Also, the device is expensive, and removal of the device is usually followed by recurrence of symptoms. Dienogest, sold under the brand name Visanne among others, is a new generation progestin medication that can be taken orally. It inhibits the development of ectopic lesions by suppressing ovarian function and the proliferation of endometrial cells. It has a highly potent progestogenic activity and lowers estradiol levels by inhibiting follicular growth [7]. Dienogest inhibits the release of gonadotropins from the pituitary gland through negative feedback regulation, resulting in reduced estrogen and increased progesterone levels in the body, factors which reduce endometrial angiogenesis, inhibit the endometrial inflammatory response, and cause ectopic endometrial tissue to metastasize. Long term use of Dienogest can also reduce the size of ectopic lesions [8]. In addition, Dienogest inhibits proliferation, induces apoptosis of uterine mesenchymal cells, reduces nerve fiber density, and reduces the expression of nerve growth factor in patients with adenomyosis [9], resulting in reduced menstrual flow and relief of symptoms [10]. The use of dienogest in the treatment of adenomyosis has only been marginally explored. In addition, the traditional Chinese herbal prescription has been widely used to treat multiple gynecological disorders. In view of this, we hypothesized that the dienogest would produce a promising outcome in patients with adenomyosis that would provide a new pharmacological alternative for conservative treatment.

## 2. Materials and Methods

### 2.1. Participants

In this retrospective study, 85 patients with adenomyosis presenting with dysmenorrhea, menorrhagia, and infertility, treated in The First Affiliated Hospital of Zhengzhou University from May 2019 to May 2021, were recruited and assigned, via the random number table method, to either an observation group (*n* = 41) or a control group (*n* = 44). The baseline characteristics of the observation group (aged 27–52 [41.44 ± 5.28] years, weighing 47–65 [55.17 ± 5.67] kg, gravidity of 1–4 [3.1 ± 1.1], and parity of 1–3 [2.2 ± 0.9]) were comparable to those of the control group (aged 28–50 [40.86 ± 5.56] years, weighing 45–65 [54.78 ± 5.10] kg, gravidity of 1–4 [2.9 ± 1.7], and parity of 1–3 [1.9 ± 0.8]) (*P* > 0.05). This study was approved by the Medical Ethics Committee of the First Affiliated Hospital of Zhengzhou University, No. #77931.

### 2.2. Inclusion and Exclusion Criteria

#### 2.2.1. Inclusion Criteria

The inclusion criteria were as follows:

1. Those with clinical symptoms that met the diagnostic criteria for adenomyosis in Obstetrics and Gynecology [11], including dysmenorrhea, menorrhagia, and infertility.
2. Those with diagnosis confirmed by either Carcinogenic Antigen 125 (CA-125) assay or imaging.
3. Those who refused to undergo hysterectomy.
4. Those with no allergies or contraindications to the drugs used in this study.
5. Those with a normal ovarian function.
6. Those with good cognitive function and normal communication abilities.
7. Those with a uterine volume that met the criteria for levonorgestrel extended-release system placement.
8. Those without concomitant endometriosis, adenomyoma, or endometrioma (also called ovarian chocolate cyst).

The exclusion criteria were as follows: Patients with allergies and contraindications to the drugs used in this study; those who had used hormonal drugs within the 3 months prior to enrollment; those with liver disease, endocrine, or autoimmune diseases; those with ovarian impairment, endometrial lesions, severe liver or kidney dysfunction; those who had used hormonal drugs in the 6 months prior to treatment; those with amenorrhea lasting more than 3 months; those suspected of having malignant disease following gynecological examination; and lastly, those who were unable to cooperate with the study.

### 2.3. Treatment Methods

Patients in the observation group received 2 mg of dienogest (Bayer Weimar GmbHund Co. KG, Germany, approval No. H20180090) daily. The drug was first administered on day 2 of the first menstrual cycle and was continued for 12 months. Patients in the control group had an LNG-IUS placed into the uterine cavity on day 3 to 7 of the menstrual cycle.

Shaoyao-Gancao Decoction (SGD), a traditional Chinese herbal prescription that contains of *Paeonia lactiflora Pall* (also known as peony) and *Glycyrrhiza uralensis Fisch*. ex DC (also known as licorice) in the ratio of 1 : 1 was given to the two groups, once a day for a total of 7 days.

### 2.4. Outcome Measures

The visual analogue scale (VAS) score, endometrial thickness, uterine volume, and menstrual volume of all enrolled patients were recorded before treatment and after 3, 6, and 12 months of treatment. Ultrasound examination was also done to comprehensively evaluate the treatment efficacy.

#### 2.4.1. Pain Profiles

The VAS scores [4] were used to evaluate the severity of dysmenorrhea, dyspareunia, and pelvic pain. Patients were instructed to rate their pain on a scale of 1 to 10 points. A score of 0 corresponds to no pain, that of 1–3 to mild pain, 4–6 to moderate pain, 7–9 to severe but tolerable pain, and a score 10 corresponds to severe and intolerable pain.

#### 2.4.2. Menstrual Volume

Menstrual flow was assessed using the pictorial blood loss assessment chart [12] (PBAC). The degree of blood staining in each sanitary pad during menstruation was noted (1 point for a blood stained area of less than or equal to a 1/3 of the sanitary pad, 5 points for a blood stained area between 1/3 and 3/5 of the sanitary pad, 20 points for a blood stained area that is almost equal to the total area of the sanitary pad, and a score >100 points for menstrual volume >80 ml).

#### 2.4.3. Uterine Changes

Uterine volume and endometrial thickness before treatment, and 3, 6, and 12 months after treatment were assessed by ultrasound and recorded. The uterine volume was calculated using the formula:

Uterine volume = 0.52 × longest diameter × anterior-posterior diameter × thickness The dimensions were obtained using ultrasound, and the ultrasound examinations were done 3–7 days after cessation of menstruation [13].

#### 2.4.4. Adverse Effects

The patients were followed up for 12 months, and adverse effects such as irregular vaginal bleeding, as well as its duration, were recorded.

### 2.5. Statistical Analysis

SPSS26.0 was used for data analysis. The measurement data are expressed as mean ± standard deviation ($\bar{x}$ ± *s*); independent samples *t*-test or ANOVA was used for intergroup comparison, and paired *t*-test was used for intragroup comparison before and after treatment. The count data are expressed as rates (%) and analyzed using the chi-square test. Differences were considered statistically significant, at *P* < 0.05.

## 3. Results

### 3.1. VAS Scores

Compared to the VAS scores before treatment, the VAS scores after treatment were significantly lower in both groups (*P* < 0.05). After 3, 6, and 12 months of treatment, patients receiving dienogest showed significantly lower VAS scores compared to those treated with LNG-IUS (*P* < 0.05) (Table 1).

### 3.2. Menstrual Volume

After treatment, the menstrual volume was significantly reduced in both groups (*P* < 0.05). After 3 months of treatment, the two groups showed similar decreases in menstrual volume (*P* > 0.05). After 6 and 12 months of treatment, dienogest produced significantly better control of menstrual volume than LNG-IUS (*P* < 0.05) (Table 2).

### 3.3. Uterine Volume and Endometrial Thickness

After 12 months of treatment, uterine volume reduction was insignificant in the observation group (*P* > 0.05), but significant in the control group (*P* < 0.05). The endometrial thickness was significantly reduced in both groups after treatment (*P* < 0.05), and there were no significant differences between the two groups (*P* > 0.05) (Table 3).

### 3.4. Adverse Effects

The main adverse effect during treatment in both groups was irregular vaginal bleeding. During treatment, the incidence of irregular vaginal bleeding lasting more than 6 months was lower in the observation group than in the control group (*P* < 0.05) (Table 4).

Most patients reported that the bleeding was tolerable. There were 3 patients in the observation group who came to the outpatient clinic for a review of their irregular vaginal bleeding, and the bleeding stopped after the patients were treated with 2–4 capsules of Zhikang (Approval No. Z20025043) three times daily. Apart from irregular vaginal bleeding, there were no statistically significant differences between the two groups in terms of adverse reactions such as breast distension, weight gain, hot flashes, night sweats, headache, insomnia, vaginitis, and back pain (*P* > 0.05). Only 1 patient in the observation group reported intolerable perimenopausal symptoms, which were relieved by a single course (28 d) of oral estradiol (Fentanyl, Abbott, The Netherlands, Approval No. H20150346). In the control group, there were 10 cases of LNG-IUS device dislodgement after 3 months of treatment, representing a dislodgement rate of 22.72% (Table 5).

## 4. Discussion

The results of the study showed that dienogest was more effective at relieving pain than LNG-IUS. After 3 months of treatment with dienogest, the patients' VAS score decreased from (8.76 ± 0.97) to (5.39 ± 1.07), and pain control was more stable with extended duration of treatment. Dienogest also produced better control of dyspareunia and pelvic pain, symptoms that were poorly controlled by LNG-IUS, with a significant reduction in scores from (5.24 ± 0.86) to (1.37 ± 0.66) following 12 months of treatment. These results are consistent with a randomized double-blind multicenter controlled study [14], which found that 130 patients with symptomatic adenomyosis who adhered to 2 mg/d dienogest for 52 weeks had a significant decrease in pain level scores and a decrease in the frequency of analgesic use. The pain scores decreased to (3.4 ± 1.8) at 24 weeks, and (3.8 ± 1.5) at 52 weeks, compared to baseline, indicating a more significant relief of dysmenorrhea in patients with symptomatic adenomyosis with long-term use of dienogest.

This study revealed that both forms of conservative treatment managed to control menstrual flow in patients with adenomyosis, and the efficacy of dienogest in controlling the menstrual flow was superior to that of LNG-IUS. However, during treatment with LNG-IUS, there was a risk of device dislodgement, especially during the first 3 months, which undermined the overall treatment efficacy. Thus, long-term continuous administration of dienogest outperformed LNG-IUS in reducing menstrual flow in patients with adenomyosis. In addition, LNG-IUS was effective in reducing uterine volume in patients with adenomyosis, while dienogest demonstrated a modest effect in reducing uterine volume.

The main adverse effect of both dienogest and LNG-IUS is irregular vaginal bleeding [15]. In the present study, irregular vaginal bleeding was particularly pronounced (up to 68.29%) in the first 3 months of treatment with dienogest, and irregular vaginal bleeding in the control group was mostly found within 6 months of treatment. With prolonged administration of dienogest, the frequency and the amount of vaginal bleeding gradually reduced. The rate of irregular vaginal bleeding in the observation group decreased to 7.32% after 6 months of treatment, a significant reduction when compared to the control group. This suggests that the incidence of irregular vaginal bleeding progressively decreases with longer duration of treatment with dienogest. An analysis of 61 patients with adenomyosis [16] stated that abnormal uterine bleeding occurred in 55 patients (90.16%) treated with dienogest, with symptoms improving as the duration of treatment became longer. The number of days of spot bleeding was (9.53 ± 11.30) at 4 weeks of administration, reducing to (6.25 ± 5.63) at 12 weeks of administration, and completely returning to normal (5.86 ± 5.61) at 24 weeks of administration, findings which are consistent with the ones in the present study. Another follow-up study of Asian patients with adenomyosis for up to 24 months [17] also arrived at the same conclusion. Therefore, informing patients in advance of the possible risk of irregular vaginal bleeding during the first few weeks of treatment with dienogest, and re-assuring them that such symptoms will progressively improve over time, may improve their long-term adherence to treatment. In addition to irregular vaginal bleeding, other common adverse effects noted in both groups include breast distension, weight gain, hot flashes, night sweats, nausea and vomiting. There was no significant statistical difference in the incidence of these side effects between the two groups. LNG-IUS device dislodgement occurred at a rate of 22.73%, mostly occurring within the first 3 months of device placement. This compromised the long-term application of LNG-IUS and prevented the device from producing a satisfactory therapeutic effect. All the findings are in consistent with the previous study that suggested a superior efficacy of dienogest to LNG-IUS that might be cost-effective.

We have to admit that there are some limitations to this study. First, the sample size was small; second, all participants were from a single center. All these might restrict its generalization and thus bias the results; third, the follow-up time was rather shorter and the observation indices were not comprehensive enough. Hence, ongoing studies with larger sample size, longer follow-up time, and multiple centers are warranted.

## 5. Conclusion

In conclusion, dienogest effectively alleviates dysmenorrhea, relieves pelvic pain, dyspareunia, and reduces menstrual flow in patients with adenomyosis, with few adverse effects and a high safety profile.

## Figures and Tables

**Table 1:** VAS scores before and after treatment ($\bar{x}$ ± *s*, points).

Groups	*n*	Dysmenorrhea				Pelvic pain or dyspareunia			
		Before treatment	3 months after treatment	6 months after treatment	12 months after treatment	Before treatment	3 months after treatment	6 months after treatment	12 months after treatment
Observation	41	8.76 ± 0.97	5.39 ± 1.07^*∗*^	3.17 ± 0.97^*∗*^^a^	2.61 ± 0.95^*∗*^^ab^	5.24 ± 0.86	2.93 ± 0.85^*∗*^	1.83 ± 0.75^*∗*^^a^	1.37 ± 0.66^*∗*^^ab^
Control	44	8.89 ± 0.99	6.11 ± 0.97^*∗*^	4.52 ± 1.07^*∗*^^a^	4.39 ± 0.92^*∗*^^ab^	5.39 ± 1.06	4.18 ± 0.82^*∗*^	2.74 ± 0.71^*∗*^^a^	2.61 ± 0.89^*∗*^^a^
*t* value		0.611	0.221	0.190	0.202	0.210	0.180	0.158	0.171
*Pvalue*		0.543	0.002	<0.001	<0.001	0.500	<0.001	<0.001	<0.001

^*∗*^indicates significant differences (*P* < 0.05) compared to before treatment; a indicates significant differences (*P* < 0.05) compared to 3 months of treatment; b indicates significant differences (*P* < 0.05) compared to 6 months of treatment.

**Table 2:** Menstrual volume before and after treatment ($\bar{x}$ ± *s*, ml).

Groups	*n*	Before treatment	3 months after treatment	6 months after treatment	12 months after treatment
Observation	41	171.78 ± 40.40	80.37 ± 13.77^*∗*^	48.98 ± 16.58^*∗*^^a^	48.29 ± 15.29^*∗*^^a^
Control	44	172.50 ± 36.48	81.23 ± 17.22^*∗*^	70.93 ± 24.16^*∗*^^a^	70.02 ± 22.81^*∗*^^a^
*t* value		0.086	3.398	4.526	4.244
*Pvalue*		0.931	0.800	<0.001	<0.001

^*∗*^indicates significant differences (*P* < 0.05) compared to before treatment; a indicates significant differences (*P* < 0.05) compared to 3 months of treatment; b indicates significant differences (*P* < 0.05) compared to 6 months of treatment.

**Table 3:** Uterine volume and endometrial thickness before and after treatment ($\bar{x}$ ± *s*).

Groups	*n*	Uterine volume (cm^3^)				Endometrial thickness (mm)			
		Before treatment	3 months after treatment	6 months after treatment	12 months after treatment	Before treatment	3 months after treatment	6 months after treatment	12 months after treatment
Observation	41	137.77 ± 47.88	136.32 ± 46.49	136.97 ± 46.48	135.35 ± 45.39	6.10 ± 1.89	3.93 ± 1.41^*∗*^	3.48 ± 1.20^*∗*^^a^	3.35 ± 1.01^*∗*^^a^
Control	44	125.84 ± 55.51	123.42 ± 54.65^*∗*^	116.87 ± 52.69^*∗*^^a^	87.34 ± 43.01^*∗*^^ab^	6.01 ± 2.36	4.07 ± 1.15^*∗*^	3.51 ± 0.89^*∗*^^a^	3.25 ± 0.81^*∗*^^a^
*t* value		1.058	11.054	10.809	9.588	0.198	0.279	0.228	0.199
*Pvalue*		0.291	0.246	0.067	<0.001	0.844	0.621	0.892	0.596

^*∗*^indicates significant differences (*P* < 0.05) compared to before treatment; a indicates significant differences (*P* < 0.05) compared to 3 months of treatment; b indicates significant differences (*P* < 0.05) compared to 6 months of treatment.

**Table 4:** Irregular vaginal bleeding (*n*, %).

Groups	*n*	None	0–3 months	4–6 months	Over 6 months
Observation	41	3 (7.32%)	28 (68.29%)	7 (17.07%)	3 (7.32%)

Control	44	1 (2.27%)	20 (45.45%)	13 (29.55%)	10 (22.73%)

*χ* ^2^					3.890

*Pvalue*					0.049

**Table 5:** Adverse events (*n*, %).

Groups	Breast tenderness	Weight gain	Hot flashes and night sweats	Headaches and insomnia	Vaginitis	Back pain	Device dislodgement
Observation	9	24	3	6	2	3	—
Control	6	26	4	5	4	9	10 (22.73%)
*χ* ^2^	1.010	0.003	0.088	0.201	0.574	3.021	10.561
*Pvalue*	0.315	0.959	0.766	0.654	0.449	0.082	0.001

## Data Availability

All data generated or analyzed during this study are included in this published article.
